The article "Human Umbilical Cord Mesenchymal Stem Cells Improve Premature Ovarian Failure through Cell Apoptosis of miR-100-5p/NOX4/NLRP3" was retracted in 2023. Reasons: unreliable results or conclusions; lack of ethics approval or compliance; concerns about the data; concerns about the peer review.

# Human Umbilical Cord Mesenchymal Stem Cells Improve Premature Ovarian Failure through Cell Apoptosis of miR-100-5p/NOX4/NLRP3

**DOI:** 10.1155/2022/3862122

**Published:** 2022-07-07

**Authors:** Jing Niu, Fan Yu, Xiping Luo, Shiling Chen

**Affiliations:** ^1^Department of Gynecology, Guangdong Women and Children Hospital, 511400, China; ^2^Department of Obstetrics and Gynecology, Nanfang Hospital, Southern Medical University, Guangzhou 510000, China

## Abstract

Premature ovarian failure refers to a series of symptoms of perimenopausal hot flashes, night sweats, decreased libido, vaginal dryness, insomnia, reduced menstruation, sparse hair, even amenorrhea, and even infertility before the age of 40 due to the decline of ovarian function. Premature ovarian failure is a common and difficult disease in gynecology. Its prevalence is increasing gradually, and the trend is younger. The aim of this experiment was to elucidate the role of human umbilical cord mesenchymal stem cells (HUCMSCs) in premature ovarian failure and its mechanism. HUCMSCs, KGN cells, and HEK293T cells were used in this experiment. Quantitative PCR and microarray analysis, ELISA inflammation and oxidative stress kits, RNA pull-down assay, luciferase reporter assay, proliferation assay, EDU staining, and Western blot analysis were used. In an in vitro model of premature ovarian failure, HUCMSCs attenuated inflammatory response, oxidative stress, and apoptosis. HUCMSCs ameliorated the premature ovarian failure model. The miR-100-5p expression was induced by HUCMSCs through methylation. miR-100-5p regulation influenced the role of HUCMSCs in an in vitro model of premature ovarian failure. HUCMSCs inhibited the in vitro expression of NOX4, NLRP3, and GSDMD proteins in the model. NOX4/NLRP3 signaling pathway affects the role of HUCMSCs in an in vitro model of premature ovarian failure through miR-100-5p. This experiment elucidated the role of HUCMSCs in premature ovarian failure and its mechanism, with a view to providing a clinical reference.

## 1. Introduction

Premature ovarian failure refers to a series of symptoms of perimenopausal hot flashes, night sweats, decreased libido, vaginal dryness, insomnia, reduced menstruation, sparse hair, even amenorrhea, and even infertility before the age of 40 due to the decline of ovarian function [1, 2]. At the same time, it is accompanied by the decrease of estrogen, the increase of follicle stimulating hormone, and the increase or unchanged of luteinizing hormone [3].

In recent years, mesenchymal stem cell therapy has made great progress in the field of animal experiment and clinical research [4]. Some research results have been applied in a variety of clinical trials, such as malignant tumors, autoimmune system diseases, nervous system diseases, and cardiovascular diseases [5–7]. Human umbilical cord mesenchymal stem cells (HUCMSCs) have achieved the results in the clinical treatment research of lupus nephritis, rheumatoid arthritis, diabetes, neuropathy, decompensated cirrhosis, liver failure, and other diseases [8–10].

MicroRNA (miRNA) is a kind of short chain, nonencoding, single-strand small molecule RNA with posttranscriptional regulation function discovered in recent years [11]. The research shows that miRNA is involved in the maturation and follicular development of mouse oocytes [12]. However, the role of miRNA in follicular development and atresia and its relationship with premature ovarian failure are still unclear. Many miRNAs are highly conserved, and their expression is tissue-specific, reflecting that they have important physiological functions and play an important role in the regulation of cell growth and development, including cell proliferation, differentiation, and apoptosis [13, 14]. The experiment elucidated the effect and underlying mechanism of human umbilical cord mesenchymal stem cells (HUCMSCs) in premature ovarian failure.

## 2. Materials and Methods

### 2.1. Cell Culture and Transfection

The human umbilical cord MSCs (HUCMSCs) from passages 3-7 were carry out as literature [15] and used for all the experiments. KGN cells (a human granulosa-like tumor cell line) and HEK293T cells were cultured in RPMI 1640 medium (Gibco, Carlsbad, CA, USA) supplemented with 10% fetal calf serum (FCS, Gibco, Carlsbad, CA, USA) in a humidified atmosphere of 5% CO_2_ at 37°C. Plasmids were transfected into KGN cells using Lipofectamine 2000. After transfection at 24 h, KGN cells (5 × 103 cells per well or 1 × 106 cells per well) cells were seeded in 96-well plates and cultured overnight. Then, the medium was removed and cultured with 100 *μ*L of serum-free medium of the hUCMSC-EVs (0.5, 1, 2 × 10^9^ per mL) for 48 h as cell proliferation assay or 24 h as other experiments.

### 2.2. Quantitative PCR and Microarray Analysis, ELISA Kits for Inflammation and Oxidative Stress, and RNA Pull-down Assay

Quantitative PCR and microarray analysis were was carry out as literature [16]. ELISA kits (Beyotime Institute of Biotechnology, China) were carry out as literature [16], and the absorbance value was quickly read using the microplate reader at a detection wavelength of 450 nm. RNA pull-down assay was carry out as literature [17].

### 2.3. Luciferase Reporter Assay

HEK293T cells were used to measure luciferase reporter. After 48 h transfection with miR-100-5p mimics or inhibitor, 500 ng pcDNA3.1 vector, or pcDNA3.1-NOX4 plasmid, HEK293T cells were harvested for luciferase activity assessment using a dual-luciferase reporter assay system (Promega).

### 2.4. Proliferation Assay and EdU Staining

After 48 h of transfection, a total of approximately 2 × 10^3^ cells/well was seeded in 96-well plate. After culturing at indicated time (0, 6, 12, 24, and 48 day), the cellular proliferation was detected using CellTiter-Glo Luminescent Cell Viability Assay (Promega, Madison, WI, U.S.A.) according to manufacturer's instructions. EdU (10 mM) was added to each well, and cells were fixed with 4% formaldehyde for 30 min. After washing, EdU was detected with Click-iTR EdU Kit, and images were visualized using fluorescent microscope (Olympus).

### 2.5. Western Blot Analysis

Western blot analysis was carried out literature [18]. The membrane was incubated with anti-NOX4 (ab133303, 1 : 1000, Abcam), anti-NLRP3 (ab263899, 1 : 1000, Abcam), and anti-*β*-actin antibody (ab8226, 1 : 5000, Abcam) at 4°C overnight. Membrane was incubated with the secondary antibody for 2 hours at room temperature. The bound antibodies were detected using enhanced chemiluminescence (ECL) with *β*-actin used as a control.

### 2.6. Statistical Analysis

Data were analyzed with GraphPad 8.0 Software and reported as the mean ± SD. The differences between groups were analyzed using Student's *t*-test or two-way ANOVA with repeated measures followed by the Tukey post hoc test. *p* < 0.05 was considered statistically significant.

## 3. Results

### 3.1. Human Umbilical Cord Mesenchymal Stem Cells Improved Premature Ovarian Failure in Model

HUCMSCs improved cell growth in vitro model of premature ovarian failure. In vitro model, HUCMSCs promoted cell growth, increased the number of EdU cell and cell metastasis, and reduced caspase-3/9 activity levels, as shown in Figure 1.

### 3.2. HUCMSCs Reduced Inflammation, Oxidative Stress, and Cell Pyroptosis in the In Vitro Model of Premature Ovarian Failure

The experiment further examined the function of the HUCMSC in vitro model of premature ovarian failure. HUCMSCs reduced IL-1*β* and IL-1*α* levels, inhibited MDA and ROS production levels, and increased SOD, CAT, and GSH-px levels in the in vitro model of premature ovarian failure, as shown in Figures 2(a)–(2j). HUCMSCs promoted cell growth, reduced LDH activity levels, increased JC-1 disaggregation and calcein-AM/CoCl2, and decreased PI levels in the in vitro model of premature ovarian failure, as shown in Figures 2(g)–2(l).  Figure 2 shows that HUCMSCs reduced inflammation, oxidative stress, and cell pyroptosis in the in vitro model of premature ovarian failure.

### 3.3. HUCMSCs Induced miR-100-5p Expression by Methylation

The experiment evaluated the mechanism of HUCMSCs on the cell pyroptosis in vitro model of premature ovarian failure. HUCMSCs promoted the miR-100-5p expression and reduced the METTL3 and METTL14 in vitro model of premature ovarian failure, as shown in Figures 3(a)–3(c). MiR-100-5p is enriched in fraction immunoprecipitated by m6A anti-body, as shown in Figure 3(d). METTL3 and METTL14 depleted and reduced m6A methylation level of miR-100-5p in NSCLC, as shown in Figure 3(f). METTL3 or METTL14 decreases miR-100-5p expression levels, as shown in Figure 3(g), suggesting that m6A methylation reduced the stability of miR-100-5p. Figure 3 shows that HUCMSCs induced the miR-100-5p expression by methylation.

### 3.4. The Regulation of miR-100-5p Affected the Effects of HUCMSC In Vitro Model of Premature Ovarian Failure

The experiment determined the role of miR-100-5p on the effects of the HUCMSC in vitro model of premature ovarian failure. MiR-100-5p mimics increased the expression of miR-100-5p, and sh-miR-100-5p reduced the miR-100-5p expression in vitro model, as shown in Figures 4(a)–4(e). The overexpression of miR-100-5p promoted the number of EdU cell and increased cell growth and cell metastasis in vitro model by HUCMSCs, as shown in Figures 4(b)–4(d). Downregulation of miR-100-5p reduced the number of EdU cell and inhibited cell growth and cell metastasis in vitro model by HUCMSCs, as shown in Figures 4(f)–4(h).  Figure 4 shows that the regulation of miR-100-5p affected the effects of the HUCMSC in vitro model of premature ovarian failure.

Next, the overexpression of miR-100-5p reduced IL-1*β* and IL-1*α* levels, inhibited MDA and ROS production levels, and increased SOD, CAT, and GSH-px levels in the in vitro model of premature ovarian failure by HUCMSCs, as shown in Figures 5(a)–5(j). The overexpression of miR-100-5p promoted cell growth, reduced LDH activity levels, increased JC-1 disaggregation and calcein-AM/CoCl2, and decreased PI levels in the in vitro model of premature ovarian failure by HUCMSCs, as shown in Figures 5(g)–5(l).

Downregulation of miR-100-5p increased IL-1*β* and IL-1*α* levels, promoted MDA and ROS production levels, and decreased SOD, CAT, and GSH-px levels in the in vitro model of premature ovarian failure by HUCMSCs, as shown in Figures 5(a)–5(j). Downregulation of miR-100-5p reduced cell growth, increased LDH activity levels, decreased JC-1 disaggregation and calcein-AM/CoCl2, and increased PI levels in the in vitro model of premature ovarian failure by HUCMSCs, as shown in Figures 5(g)–5(l).  Figure 5 shows that the regulation of miR-100-5p affected the effects of HUCMSCs on inflammation, oxidative stress, and cell pyroptosis in vitro model of premature ovarian failure.

### 3.5. NOX4/NLRP3 Signaling Pathway Affected the Effects of HUCMSCs In Vitro Model of Premature Ovarian Failure by miR-100-5p

To further investigate the mechanism of HUCMSCs on premature ovarian failure by miR-100-5p, we analyzed the effects of HUCMSC regulated signaling pathway in model of premature ovarian failure. NOX4/NLRP3 signaling pathway might be one target spot for HUCMSCs on premature ovarian failure, as shown in Figures 6(a)–6(c). Meanwhile, HUCMSCs reduced NOX4 mRNA expression, and sh-miR-100-5p increased the NOX4 mRNA expression in vitro model, as shown in Figure 6(d). HUCMSCs reduced the effects of sh-miR-100-5p on the NOX4 mRNA expression in vitro model, as shown in Figure 6(d). Meanwhile, HUCMSCs reduced the NOX4 mRNA expression in vitro model, as shown in Figure 6(e). Luciferase reporter assay illustrated that NOX4 wild type (WT) closely correlated with miR-100-5p by HUCMSCs, as shown in Figure 6(f). The WT and corresponding mutant (Mut) were constructed targeting the miR-100-5p in vitro model, as shown in Figure 6(f). The overexpression of miR-100-5p reduced the NOX4 mRNA expression in vitro model by HUCMSCs, as shown in Figure 6(g). Downregulation of miR-100-5p increased the NOX4 mRNA expression in vitro model by HUCMSCs, as shown in Figure 6(h). HUCMSCs suppressed NOX4, NLRP3, and GSDMD protein expression levels in the in vitro model, as shown in Figures 7(a)–7(c). The overexpression of miR-100-5p reduced the effects of HUCMSCs on NOX4, NLRP3, and GSDMD protein expression levels in the in vitro model, as shown in Figures 7(d)–7(f). Downregulation of miR-100-5p increased the effects of HUCMSCs on NOX4, NLRP3, and GSDMD protein expression levels in the in vitro model, as shown in Figures 7(g)–7(i). Figure 6 shows that NOX4/NLRP3 signaling pathway affected the effects of the HUCMSC in vitro model of premature ovarian failure by miR-100-5p.

## 4. Discussion

Premature ovarian failure refers to the premature decline of ovarian function, that is, the state of low estrogen and high gonadotropin before the age of 40 [19]. The pathogenesis of premature ovarian failure is not clear, involving chromosome abnormalities, gene mutations, autoimmune diseases, granulosa cell, and mitochondrial abnormalities [12]. Traditional Chinese medicine and other treatment mechanisms also involve many aspects, such as reproductive endocrine hormone level, immune function, related signal transduction pathways, granulosa cell apoptosis, and noncoding RNA [20]. In this study, HUCMSCs promoted cell growth, increased the number of EdU cell and cell metastasis, and reduced caspase-3/9 activity levels in the in vitro model. Shareghi-Oskoue et al. showed that HUCMSCs could treat premature ovarian failure [21]. These data indicated that HUCMSCs promoted cell recovery to improve premature ovarian failure.

Ovary is the female reproductive organ [22]. Its main function is to maintain the function of the female reproductive system and the secretion of hormones [23]. The imbalance of free radical metabolism caused by endemic fluorosis and the damage of organ function caused by the accumulation of a large number of oxidative stress products have always been a hot issue for researchers [23]. Oxidative stress injury will promote the production of inflammatory factors [24]. The level of oxidative stress has been used as a biological marker of premature aging [25]. In this study, we showed that HUCMSCs reduced inflammation, oxidative stress, and cell pyroptosis in vitro model of premature ovarian failure. Nie et al. reported that hUCMSCs attenuated apoptosis and oxidative damage and in type 2 diabetes mellitus [26]. These results suggested HUCMSCs reduced inflammation and oxidative stress to inhibit cell pyroptosis in model of premature ovarian failure.

As a common endogenous single stranded noncoding small RNA molecule, miR-100-5p participates in the pathophysiological processes of many diseases, including inhibiting cell apoptosis and promoting cell proliferation [27, 28]. Similarly, our study validated HUCMSC-induced miR-100-5p expression by methylation. Gao et al. demonstrated that miR-100-5p in HUCMSCs inhibits cell progression and inflammatory response in eosinophils, thereby alleviating atherosclerosis progression [29]. These findings showed the HUCMSC inflammation, oxidative stress, and cell pyroptosis by the promotion of miR-100-5p.

The main biological function of NOX family proteins is to produce ROS, which can maintain the normal physiological activities of cells [30]. Oxidative stress caused by increased ROS in the body is related to a variety of diseases. The research on the pathogenic mechanism of the NOX family is of great significance in the prevention, diagnosis, and treatment of clinical diseases. Here, we confirmed that HUCMSCs suppressed NOX4 signaling pathway in model of premature ovarian failure by miR-100-5p. Zhong et al. showed that HUCMSCs protected against DOX-induced heart failure through miR-100-5p/NOX4 pathway [31]. These data indicated that HUCMSCs suppressed NOX4 expression by miR-100-5p in model of premature ovarian failure.

NLRP3 can promote the secretion of proinflammatory cytokines, aggravate cell damage, and induce cell death [32, 33]. Inhibiting NLRP3 inflammatory signal can reduce inflammatory response and protect tissues, promote the release of anti-inflammatory cytokine IL-10 and proinflammatory cytokine IL-21 levels in serum, improve the inflammatory response of ovary, and reduce the inflammatory injury of follicle and the decline of ovarian reserve function [20–34]. This study showed that the HUCMSCs suppressed NOX4, NLRP3, and GSDMD protein expression levels in the in vitro model. Yuan et al. revealed that HUCMSCs inhibit nucleus pulposus cell pyroptosis through METTL14/NLRP3 [1, 35]. These findings suggested that HUCMSCs reduced cell pyroptosis to improve premature ovarian failure through the inhibition of NOX4/NLRP3.

## 5. Conclusion

In conclusion, HUCMSCs reduced cell pyroptosis to improve premature ovarian failure through the inhibition of NOX4/NLRP3 by methylation of miR-100-5p. This study provided a new mechanism for the understanding of the HUCMSCs which improve premature ovarian failure and indicated novel target for premature ovarian failure treatment. This infers that HUCMSCs are potential targets to be used in the treatment of premature ovarian failure.

## Figures and Tables

**Figure 1:** Human umbilical cord mesenchymal stem cells improved premature ovarian failure in model cell growth (a), the number of EdU cell (b), cell metastasis (c), and caspase-3/9 activity levels (d, e). Control: control group; low/med/high: low/med/high of the HUCMSC group. ^∗∗^*p* < 0.01 compared with the control group.

**Figure 2:** HUCMSCs reduced inflammation, oxidative stress, and cell pyroptosis in vitro model of premature ovarian failure IL-1*β* and IL-1*α* levels (a, b), ROS production levels (c), MDA level (d), SOD (e), CAT (f) and GSH-px (j) levels, cell growth (g), LDH activity levels (h), JC-1 disaggregation (i), PI levels (k), and calcein-AM/CoCl2 (l). Control: control group; low/med/high: low/med/high of the HUCMSC group. ^∗∗^*p* < 0.01 compared with the control group.

**Figure 3:** HUCMSCs induced the miR-100-5p expression by methylation miR-100-5p expression (a), METTL3 and METTL14 mRNA expression (b, c), RIP-PCR assays performed by using m6A anti-body (d), depletion either METTL3 or METTL14 led to m6A modification level (e), and si-METTL3 or si-METTL14 resulted in downregulation of miR-100-5p level (f). Control: control group; low/med/high: low/med/high of the HUCMSC group. METTL3 or METTL14: METTL3 upregulation or METTL14 upregulation group. ^∗∗^*p* < 0.01 compared with control or negative control group.

**Figure 4:** The regulation of miR-100-5p affected the effects of the HUCMSC in vitro model of premature ovarian failure MiR-100-5p (a), the number of EdU cell (b), cell metastasis (c), cell growth in vitro model by overexpression of miR-100-5p (d), MiR-100-5p (e), the number of EdU cell (f), cell metastasis (g), and cell growth in vitro model by downregulation of miR-100-5p (h). Vector: negative control group; miR-100-5p: overexpression of miR-100-5p group; sh-nc: sh-negative control group; sh-miR-100-5p: downregulation of miR-100-5p group; HUCMSCs: HUCMSC group; ^∗∗^*p* < 0.01 compared with vector or sh-negative control group.

**Figure 5:** The regulation of miR-100-5p affected the effects of HUCMSCs on inflammation, oxidative stress, and cell pyroptosis in vitro model of premature ovarian failure IL-1*β* and IL-1*α* levels (a, b), ROS production levels (c), MDA level (d), SOD (e), CAT (f), and GSH-px (j) levels, cell growth (g), LDH activity levels (h), JC-1 disaggregation (i), PI levels (k), and calcein-AM/CoCl2 (l). Vector: negative control + HUCMSC group; miR-100-5p: overexpression of miR-100-5p + HUCMSC group; sh-nc: sh-negative control + HUCMSC group; sh-miR-100-5p: downregulation of miR-100-5p + HUCMSC group; ^∗∗^*p* < 0.01 compared with vector or sh-negative control group.

**Figure 6:** NOX4/NLRP3 signaling pathway affected the effects of the HUCMSC in vitro model of premature ovarian failure by miR-100-5p heat map and combine sample correlation (a), volcanic map (b), result analysis (c), NOX4 mRNA (d, e), luciferase reporter levels and KLF13 constructed targeting miR-100-5p (f), and NOX4 protein expression (g, h). Control: control group; low/med/high: low/med/high of the HUCMSC group. Vector: negative control group; miR-100-5p: overexpression of miR-100-5p group; sh-nc: sh-negative control group; sh-miR-100-5p: downregulation of miR-100-5p group; HUCMSCs: HUCMSC group; ^∗∗^*p* < 0.01 compared with vector or sh-negative control group.

**Figure 7:** NOX4/NLRP3 protein expression in NOX4, NLRP3, and GSDMD protein expression levels in the in vitro model by HUCMSCs; HUCMSCs promoted NOX4, NLRP3, and GSDMD protein expression (a)–(c), NOX4, NLRP3, and GSDMD protein expression levels in the in vitro model by overexpression of miR-100-5p + HUCMSCs (d)–(f), and NOX4, NLRP3, and GSDMD protein expression levels in the in vitro model by downregulation of miR-100-5p + HUCMSCs (g)–(i). Control: control group; low/med/high: low/med/high of the HUCMSC group. Vector: negative control group; miR-100-5p: overexpression of the miR-100-5p group; sh-nc: sh-negative control group; sh-miR-100-5p: downregulation of the miR-100-5p group; HUCMSCs: HUCMSC group; ^∗∗^*p* < 0.01 compared with vector or sh-negative control group.

## Data Availability

The simulation experiment data used to support the findings of this study are available from the corresponding author upon request.
